The article "Artificial photoactive chlorophyll conjugated vanadium carbide nanostructure for synergistic photothermal/photodynamic therapy of cancer" was retracted in 2023. Reasons: duplicated images; overlap with earlier publications; original data or images not available; unreliable data.

# Artificial photoactive chlorophyll conjugated vanadium carbide nanostructure for synergistic photothermal/photodynamic therapy of cancer

**DOI:** 10.1186/s12951-022-01331-x

**Published:** 2022-03-09

**Authors:** Huiting Lu, Shah Zada, Songsong Tang, Cheng Yaru, Wei Wei, Qiao Yuchun, Qiqi Yang, Jinya Du, Pengcheng Fu, Haifeng Dong, Xueji Zhang

**Affiliations:** 1 School of Chemistry and Biological Engineering, University of Science & Technology Beijing, 0 Xueyuan Road, Beijing, 100083 People’s Republic of China; 2 Marshall Laboratory of Biomedical Engineering, Research Center for Biosensor and Nanotheranostic, School of Biomedical Engineering, Shenzhen University, Guangdong, 518060 People’s Republic of China; 3 Beijing Key Laboratory for Bioengineering and Sensing Technology, Research Center for Bioengineering and Sensing Technology, School of Chemistry and Bioengineering, University of Science & Technology Beijing, Beijing, 100083 People’s Republic of China; 4 State Key Laboratory of Marine Resource Utilization in South China Sea Hainan University, 58 Renmin Avenue, Meilan District, Haikou, Hainan Province 570228 People’s Republic of China

**Keywords:** Optically active nanostructures, Photothermal therapy, Photodynamic therapy, Chlorophyll, Vanadium carbide

## Abstract

Optically active nanostructures consisting of organic compounds and metallic support have shown great promise in phototherapy due to their increased light absorption capacity and high energy conversion. Herein, we conjugated chlorophyll (Chl) to vanadium carbide (V_2_C) nanosheets for combined photodynamic/photothermal therapy (PDT/PTT), which reserves the advantages of each modality while minimizing the side effects to achieve an improved therapeutic effect. In this system, the Chl from *Leptolyngbya JSC-1* extracts acted as an efficient light-harvest antenna in a wide NIR range and photosensitizers (PSs) for oxygen self-generation hypoxia-relief PDT. The available large surface of two-dimensional (2D) V_2_C showed high Chl loading efficiency, and the interaction between organic Chl and metallic V_2_C led to energy conversion efficiency high to 78%. Thus, the Chl/ V_2_C nanostructure showed advanced performance in vitro cell line killing and completely ablated tumors in vivo with 100% survival rate under a single NIR irradiation. Our results suggest that the artificial optical Chl/V_2_C nanostructure will benefit photocatalytic tumor eradication clinic application.

**Graphical Abstract:**

**Supplementary Information:**

The online version contains supplementary material available at 10.1186/s12951-022-01331-x.

## Introduction

Cancer is a stressful and dangerous disease because of the maximum occurrence rate in humans and high mortality [1]. In the past few years, besides traditional surgery, chemotherapy, and radiotherapy, massive attention has been devoted to discovering non-invasive safe and suitable alternative approaches for this critical disease breakthrough [2]. Non-invasive and highly-selective phototherapy typically carried out in photodynamic therapy (PDT) and photothermal therapy (PTT) hold great promise in cancer treatments [3]. PDT is a promising tumor ablative therapeutic approach in the field of oncology [4]. It depends on the laser-induced ability of photosensitizers (PSs) to transfer energy to oxygen dissolved in the tumor environment to generate cytotoxic singlet oxygen (O^1^_2_), which enabled successively causing cell death and mortality of immediate tumor tissues [5]. However, the PDT efficiency of solid tumors is mostly unsatisfying by issues involving the hydrophobic and hypoxic tumor microenvironment (TME) [6] and limited light penetrability [7].

The article "Artificial photoactive chlorophyll conjugated vanadium carbide nanostructure for synergistic photothermal/photodynamic therapy of cancer" was retracted in 2023. Reasons: duplicated images; overlap with earlier publications; original data or images not available; unreliable data.

Photothermal therapy (PTT) has been considered a progressively advanced, safe, and promising therapeutic approach for cancer [4]. Near-infrared (NIR) irradiation is regularly applied to produce heat for hyperthermia of tumor spots without damaging normal tissue cells [3]. The photothermal conversion agent (PTCA) absorbs light energy as a source and converts it into heat, which significantly determines nanomaterial-based PTT performance [8]. Two correlated procedures can clearly and quantitatively define the photothermal ability of PTCA [9]. The first procedure mainly concentrated on the absorption of NIR light to obtain energy from irradiation. The value could be fixed by the molar elimination quantity of the materials [10]. The second procedure relates to the energy transformation pathways from the absorbed light to heat, generally related to photothermal conversion proficiency [11]. Thus, the PTCA agents performed a crucial role in manipulating the photothermal effect of their practical/clinical applications [12]. The PTCA agents with superior NIR light absorption capacity and reduced non-thermal radiative conversions are still essential [13].

PTT/PDT synergistic therapy of cancers has attracted great interest. In comparison with a single treatment, the PTT/PDT therapy strategies inherited the advantages of each modality while minimizing its side effects, which thus have resulted in a significantly enhanced therapeutic effect. The appropriate heating by PTT enabled increased blood flow and improved oxygen supply for enhanced PDT, and hyperthermia can also improve PDT-induced damages. PDT can disturb TME conditions and result in increased heat sensitivity of cancer cells. To date, many types of nanomaterials have been employed for dual-modality PTT/PDT [14, 15]. The development of optically active nanostructures with extraordinary physicochemical properties to conduct coinciding synergistic PDT/PTT treatment under irradiation is urgently needed [16].

The article "Artificial photoactive chlorophyll conjugated vanadium carbide nanostructure for synergistic photothermal/photodynamic therapy of cancer" was retracted in 2023. Reasons: duplicated images; overlap with earlier publications; original data or images not available; unreliable data.

Herein, we fabricated a Chl/V_2_C optically active nanostructures by assembling Chl to V_2_C nanosheets (NSs) to realize synergistic PDT/PTT with improved therapeutic effect. The Chl from *Leptolyngbya JSC-1* extract enabled efficient light harvest in a wide NIR range and implemented oxygen self-generation for hypoxia-relief PDT. The two-dimension V_2_C provided a large surface for Chl loading. The interaction between organic Chl and metallic V2C results in high energy conversion and highly-effective photothermal conversion efficiency for PTT. Under NIR irradiation, the Chl/V_2_C nanostructure showed advanced anticancer performance in vitro cell line killing and tumor ablation in vivo. (Scheme 1). The chlorophyll (Chl) is a green pigment and light-sensitive substance. The chemical formula of (Chl) is C_55_H_72_MgN_4_O_5_. It is automatically activated after the NIR light strikes. It generates a special kind of oxygen molecule or ROS that kills the tumor cells (Additional file 1: Scheme S1). The artificial optical Chl/V_2_C nanostructure holds excellent potential in synergistic PDT/PTT.

**Scheme 1:** Schematic illustration of Chl/V_2_C nanostructure for synergistic PTT/PDT. Note Because chl is very strong light sensitive and having high potential to convert light energy to thermal energy

## Materials and methods

### Instrument

Transmission electron microscopy (TEM), high-resolution transmission electron microscopy (HRTEM) and energy dispersive X-ray spectroscopy spectra (EDX) were performed on a JEM-2100F transmission electron microscope (HITACHI, Japan). UV–Vis absorption spectra were collected by a UV-3600 Shimadzu UV–Vis spectrometer (Shimadzu, Japan). Fourier transform infrared spectroscopy (FTIR) was performed using a Nicolet 6700 FT-IR spectrometer. The oxygen meter was utilized to measure oxygen concentration generation in solutions (JPBJ-606, INESA, and China). The temperature and thermal images were recorded on an infrared thermal imaging instrument (Fluke TiS65, USA). The Dynamic light scattering (DLS) analysis was used to obtain the size of the synthesized nanosheet (Malvern Instruments Zetasizer Nano ZS90). The confocal laser scanning microscopy (CLSM) images were acquired on the FV1200 microscope (Olympus, Japan).

### Extraction of Chl

Twenty grams of *Leptolyngbya* JSC-1 were milled in 100 mL of liquid nitrogen with a mortar and pestle for 5 min. The extract was gently shifted to a fresh bottle and washed the crusher thoroughly with acetone. The volume was adjusted exactly to 500 mL by adding acetone to the glass bottle, followed by incubation for 8 h. Then, the extract was filtered using Millipore membrane (0.2 µm pore size) to eliminate contaminations. After filtration, the solution was centrifuged for 10 min at 1500 rpm to collect the supernatant of the solution. The extracted Chl was compared with standard Chl under a UV spectrophotometer [17].

The article "Artificial photoactive chlorophyll conjugated vanadium carbide nanostructure for synergistic photothermal/photodynamic therapy of cancer" was retracted in 2023. Reasons: duplicated images; overlap with earlier publications; original data or images not available; unreliable data.

### Green synthesis of V_2_C NSs

The V_2_C NSs were synthesized according to our previous study [18]. The powder of V_2_AlC (roughly 100 mg) mixed with a 20 mL solution of algae extract was added into the water with a final volume of 100 mL and stirred for one day at room temperature. The resultant mixture was carefully washed with water and ethanol by centrifugation. The pellet was dispersed in 50 mL of water and stirred for an additional 1 day at room temperature. Then V_2_C NSs were collected by centrifuging at 5000 g for 10 min and washed thrice with ethanol and water to remove the other remains.

### Fabrication of Chl/V_2_C NSs

20 µL Chl was mixed with V_2_C (5 mg/mL) and sonicated for 30 min to fully incorporate the Chl on the surface of the V_2_C NSs. The resulting Chl/V_2_C was washed three times. The loaded Chl molecules on V2C were investigated with UV–Vis spectroscopy at different intervals of time [19].

### Photothermal performance of the Chl/V_2_C

1 mL Chl/V_2_C aqueous solution with different concentrations (0, 5, 10, 20, 40, and 80 µg / mL, where 0 is the control group) were examined in a quartz cuvette that exposed to an 808 nm laser (0.48 W cm^−2^) for 5 min, following by 10 min natural cooling. To examine the photothermal stability of the samples, repeat five times the heating and cooling cycle. The temperature was observed using a thermocouple at various an interval [18].

### Cell cytotoxicity evaluation

The MCF-7 cells were cultured in Gibco Dulbecco's Modified Eagle Medium (DMEM) medium containing 1% penicillin/streptomycin (P/S) and 10% fetal bovine serum (FBS) at 37 °C and 5% CO_2_ in a moist atmosphere. Initially, the MCF-7 cells were seeded in a 96-wells plate for 24 h at a 1 × 10^4^ density of cells per well. The cells were treated with control, V_2_C, Chl, and Chl/V_2_C in different concentrations (0, 10, 20, 40, 80, 160 µg / mL) for 4 h. Consequently, the new media were replaced and kept for 24 h again. 10 μL of microculture tetrazolium assay solution was added to each well (5 mg mL^−1^ phosphate-buffered saline (PBS) (pH 7.4,10 mM). After the incubation for another 4 h, the cell viability was determined by a microplate reader at 492 nm. For CLSM images, cells were cultured for 24 h. Then the media were replaced with fresh media containing PBS (pH 7.4,10 Mm), V_2_C, Chl, and Chl/V_2_C and incubated for 4 h. Afterward, the cells were stained with dual dyes PI and Cancelin for 10 min and then washed with PBS (pH 7.4,10 Mm) before examining them under a CLSM, according to our previous report [15, 18, 20, 21].

The article "Artificial photoactive chlorophyll conjugated vanadium carbide nanostructure for synergistic photothermal/photodynamic therapy of cancer" was retracted in 2023. Reasons: duplicated images; overlap with earlier publications; original data or images not available; unreliable data.

### Singlet oxygen generation capability of Chl/V_2_C

The DCFH-DA probe was used to measure the ^1^O_2_ generation ability of Chl, V_2_C and Chl/V_2_C under NIR laser irradiation. 5 μL of DCFH-DA was added into the solution of Chl (1 mL, 80 μg/ mL), V_2_C nanosheet (1 mL, 80 μg/ mL) and Chl/V_2_C (1 mL, 80 μg/ mL) irradiated with a 670 nm laser (0.48 W cm^−2^) for 5 min. The fluorescence of DCFH-DA at 410 nm was continuously recorded for 10 min and the ^1^O_2_ dramatic yield was calculated [21].

### In Vitro PTT and PDT therapeutic efficacy

The cells were seeded in confocal dishes for 24 h with a density of 1 × 10^4^ cells per well. Cells were treated as follows: PBS (phosphate buffer solution) (pH 7.4,10 mM), Laser (670 & 808 nm), V_2_C (1 mL, 80 μg/ mL), Chl (1 mL, 80 μg/ mL), Chl/V_2_C(1 mL, 80 μg/ mL), Chl/V_2_C (1 mL, 80 μg/ mL) + 670 nm laser, Chl/V_2_C(1 mL, 80 μg/ mL) + 808 nm laser, Chl/V_2_C(1 mL, 80 μg/ mL) + 670 & 808 nm laser (0.48 W cm^−2^). After exposure, the culture media were removed and the cells were thoroughly washed with PBS. For CLSM imaging, all groups were stained using dual dyes Calcein-AM and PI. For intracellular ^1^O_2_ generation measurement, the cells were incubated in confocal cultured dishes for 24 h and treated as aforementioned for 4 h. Afterward, the media were replaced with fresh DMEM and incubated for another 12 h. Cells were stained with SOSG (2 μL) and Hoechst 33342 for 10 min (2 μL, 2 × 10^−3^ m), and then CLSM was used for observing cells.

### In vivo PTT/PDT

Four to five-week-old Balb/c nude female mice were purchased from Beijing Vital River Laboratory Animal Technology Co, Ltd. All animal experimentations were done following the recommended protocol. 100 μL of PBS (pH 7.4,10 mM) containing 2 × 10^6^ MCF-7 cells were subcutaneously inoculated into the back of every mice. The mice were randomly arranged into 8 groups (each containing five mice) when the tumor volume reached 200 mm^3^ (*V* = width^2^ × length/2). The drug were intravenously injected/treated into the tail vein of mice as follows: (1) PBS (pH 7.4,10 mM), (2) Laser (670 & 808 nm), (3) Chl/V_2_C (1 mL, 80 μg/ mL) (4) Chl (1 mL, 80 μg/ mL) + 670 nm laser, (5) V_2_C (1 mL, 80 μg/ mL) + 808 nm laser, (6) Chl/V_2_C (1 mL, 80 μg/ mL) + 670 nm laser, (7) Chl/V_2_C (1 mL, 80 μg/ mL) + 808 nm laser and (8) Chl/V_2_C (1 mL, 80 μg/ mL) + 670 & 808 nm laser irradiation for 5 min (0.48 W cm^−2^), respectively. The tumor volume and body weight were measured at intervals of 3 days for 2 weeks. For histological analysis, principal organs and tumor tissues were collected [18].

The article "Artificial photoactive chlorophyll conjugated vanadium carbide nanostructure for synergistic photothermal/photodynamic therapy of cancer" was retracted in 2023. Reasons: duplicated images; overlap with earlier publications; original data or images not available; unreliable data.

### The blood circulation and biodistribution of Chl/V_2_C NSs

MCF-7 cells were introduced to mice follow the above method. The MCF-7 tumors mice were treated intravenously with Chl/V2C NSs (10 mg/kg). After intravenous injection the (50 µL) blood samples were collected from the eye socket at 0.5, 1, 3, 6, and 12 h (*n* = 5) of each interval respectively. The collected blood sample were treated with H_2_O_2_/HNO_3_ solution (1:3) and Mg/V concentrations were measured by ICP-MS, which devoted Chl/V_2_C NSs. The tumor-bearing mice were sacrificed after 12 h of injection. To evaluate the distribution of Chl/V_2_C NSs in the various tissue/organs, such like (heart, liver, spleen, lung, kidney, and tumor were collected, weighed, and dissolved with H_2_O_2_/HNO_3_ mixture solution (1:3), and measured the Mg/V concentration using ICP-MS and Mg/V concentrations were measured by ICP-MS, which devoted Chl/V_2_C NSs. Under license no, all animal protocols were approved by the institutional animal ethics review committee of the Peaking University Health Science Center. SYXK (京)-2016–0010.

### In vitro hypoxic investigation

The cells were incubated in PBS and DMEM media containing Chl/V_2_C (1 mL, 80 μg/ mL) in confocal dishes along with or without laser 670 (0.48 W cm^−2^) irradiation for 10 min individually, keeping for 4 h. Afterward, all the groups were shifted to a translucent box and exposed to N_2_ atmosphere. Successively, the cells media were replaced with fresh media and incubated for 24 h. Then cells were examined under the confocal microscope [21].

### Tumour model hypoxia measuring

Again MCF-7 cell inserted intravenously to mice like above. And growth of tumour was monitored until it reached the size of 200 mm^3^ (*V* = width^2^ × length/2). Then, Chl/V_2_C SNs (10 mg/kg-1) was injected into the mice via the tail vein After 24 h, the mice were irradiated with a 670 & 808 nm laser irradiation for 5 min (0.48 W cm^−2^) Then, the mice were injected intraperitoneally with saline solution containing pimonidazole hydrochloride (60 mg/kg). After 1 h, the mice were scarified and the tumor tissues were harvested. For immunofluorescence staining, the tumor hypoxia regions were labeled with FITC-MBb1 (antipimonidazole antibody). Next, the slices were stained with an anti-FITC secondary antibody and to determine the % hpoxia were measured subsequent analyses by using CLSM [21].

The article "Artificial photoactive chlorophyll conjugated vanadium carbide nanostructure for synergistic photothermal/photodynamic therapy of cancer" was retracted in 2023. Reasons: duplicated images; overlap with earlier publications; original data or images not available; unreliable data.

### Statistical analysis

The data were analyzed and demonstrated as the mean, standard deviations (SD), and experimental triplicates for statistical significance.

## Results and discussion

### Characterization of Chl/V_2_C

The UV–Vis spectrum of extracted Chl showed two characteristic solid peaks at 433 and 662 nm, similar to the standard sample of Chl (Additional file 1: Fig. S1A), which confirmed the successful extraction of Chl from algae extracts [22]. The functionalization of V_2_C NSs with Chl appeared two new strong peaks at 453 and 735 nm (Additional file 1: Fig. S1B). The red-shift of both peaks compared to the Chl resulted from the interaction between the metallic V_2_C NSs and organic Chl. The intensity of the peaks increased along with the increase of incubated time until 15 min (Additional file 1: Fig. S1C), and the maximum loading efficiency was calculated to 10 µg, suggesting good loading efficiency. The V_2_C NSs were successfully exfoliated into a single-layer structure [18]. The V_2_C, Chl and Chl/V_2_C Zeta potential anlysis were investgated in (Additional file 1: Fig. S2) They showed a narrow size distribution with a mean size of 50–70 nm (Fig. 1A). The fast Fourier transform (FFT) pattern indicated a hexagonal structure of the crystalline lattice of V_2_C NSs, confirming the well-crystallized nature and successful synthesis of V_2_C NSs (Fig. 1B). The surface V_2_C NSs was decorated with many Chl nanoparticles with a size of about 30 nm after modifying Chl (Fig. 1C). The zeta potential of Chl/V_2_C NS showed a significant decrease to -19.5 mV compared with pure V_2_C NSs after negatively charged Chl loading (Fig. 1D). The remarkable changes in the surface charges advocated the successful assembly of Chl/V_2_C NS. The elemental mapping of V_2_C NSs, Chl and Chl/V_2_C NSs confirmed the successful fabrication of Chl/V_2_C NSs (Fig. 1E and Additional file 1: Fig. S3). The FT-IR spectra of Chl/V_2_C NSs presented the characteristic peaks derived from both Chl and (Fig. 1F), validating further the successful assembly of Chl/V_2_C NSs.

**Fig. 1:** **A** TEM images and **B** FFT pattern of V_2_C, **C** TEM images of Chl/V_2_C, **D** Zeta potential, **E** Element mapping and **F** FTIR of Chl, V_2_C, and Chl/V_2_C

### Photothermal performance and ROS generation ability of Chl/V_2_C SNs

The O_2_ generation ability of Chl/V_2_C NSs under NIR irradiation through water splitting was validated in (Fig. 2A), which was beneficial to relieve hypoxic tumor microenvironment (TME) for enhanced PDT performance [23]. The ROS production of Chl/V_2_C NSs was investigated using a fluorescent probe, where the 2, 7-Dichloro fluorescein diacetate (DCFH-DA) probes were oxidized to produce green fluorescence (Fig. 2B). The intensity of DCFH-DA fluorescence displayed a constant increase in Chl/V_2_C NSs solution under a 670 nm laser irradiation (0.48 W/cm^2^) for 10 min. Enhanced ROS generation ability of Chl/V_2_C was observed compared to V_2_C and Chl (Fig. 2C). The ROS production was further characterized by (ESR) electron spin resonance. It demonstrated that Chl/V_2_C improved generation ability for several types of ROS species, including ^1^O_2_, ·OH and·O_2_^−^ (Fig. 2D–F). The advanced ROS generation ability was resulted from the interaction between the V_2_C NSs and Chl to enhance photogenerated electron sets parting efficiency at the edge. The chlorophyll has 2-carboxylic acid moiety, in which N-linked to a pyridine dicarboxylic acid group through an acetyl group. The conjugated bonds in these ring systems are responsible for absorbing visible light in the green region. As seen from its structure, it has several carboxylic acid groups, promising good dipole interactions with V_2_C SNs and strong attaching, and a good choice for photo-sensitizer [20]. Chl/V2C NSs' good conductivity at the border maintained the electron transmission and reserved the recombined electron [21, 24].

The article "Artificial photoactive chlorophyll conjugated vanadium carbide nanostructure for synergistic photothermal/photodynamic therapy of cancer" was retracted in 2023. Reasons: duplicated images; overlap with earlier publications; original data or images not available; unreliable data.

**Fig. 2:** **A** O_2_ generation of Chl/V_2_C (80 µg/mL) aqueous solution under a 670 nm laser (0.48 W/cm^2^) irradiation. **B** ROS generation Chl/V_2_C (80 µg/mL) measured by DCFH-DA probe under a 670 nm laser (0.48 W/cm^2^). **C** The comparsion of ROS generation of PBS (pH 7.4,10 Mm), V_2_C, Chl and Chl/V_2_C (80 µg/mL) under a 670 nm laser irradiation (0.48 W/cm^2^) monitored by DCFH fluorescence probe. ESR spectra of V_2_C, Chl and Chl/V_2_C (80 µg/mL) under a 670 nm laser (0.48 W/cm^2^) irradiation for characterization of **D** ^1^O_2_, **E**·OH and **F**·O_2_^−^. **G** The UV–vis absorption spectra, **H** photothermal heating curves of Chl/V_2_C with various concentrations and photostability of Chl/V_2_C (80 µg/mL) irradiated by a 808 nm laser (0.8 W/cm^2^) irradiation

The Chl/V_2_C SNs presented a strong absorption in the wide NIR range (Fig. 2G), which showed a concentration-dependent increase in temperature under irradiation. The temperature of Chl/V_2_C SNs NSs (80 µg/mL) improved to 73.2 ℃. In contrast, the control temperature only increased to 29.2 ℃ under irradiation for 10 min (Fig. 2H) [18, 25]. The different ratios of Chl loading in V_2_C nanosheets were investigated. As a result, the greatest phototherapy transfer efficiency and singlet oxygen production efficiency were obtained (Additional file 1: Fig. S4). The photothermal conversion efficiency (PTCE) was measured to 78% (Additional file 1: Fig. S4) derived from the cooling curve, which was stronger to other 2D PTAs nanomaterials including MoS_2_ NSs (24.37) [26] V_2_C (47.5%)[18] Ti_3_C_2_/g-C_3_N_4_ NSs (40.8%) [21] and Ti_3_C_2_@Met@CP (59.6%)[27]. The high PTCE was because of Chl/V_2_C enhanced light absorption capacity and high energy conversion efficiency [28]. The Chl/V_2_C NSs also demonstrated excellent photothermal stability under a 808 nm laser (0.48 W/cm^2^) irradiation for 5 min, with on & off laser cycles for five times (Fig. 2I).

The article "Artificial photoactive chlorophyll conjugated vanadium carbide nanostructure for synergistic photothermal/photodynamic therapy of cancer" was retracted in 2023. Reasons: duplicated images; overlap with earlier publications; original data or images not available; unreliable data.

### In vitro anticancer performance of Chl/V_2_C NSs and their biosafety analysis

MTT was used to investigate the cytotoxicity of Chl/V_2_C NSs, the viability of MCF-7 cells were still beyond 98% even at a concentration higher than 160 µg/mL, validating the little cytotoxicity of Chl/V_2_C NSs compared to control, Chl and V_2_C (Fig. 3A), [29] which also be validated by the Calcein-AM/PI dual-stained analysis (Fig. 3B). The low cytotoxicities of Chl/V_2_C NSs towards HeLa and A549 were also validated (Additional file 1: Fig. S6). These results concluded the excellent biocompatibility of Chl/V_2_C NSs because chlorophyll is a natural green active pigment and Chl/V_2_C biocompatibility is more superior to other reported materials such as V_2_C, Mo_2_C, Ti_2_C and Ti_3_C. As shown in (Fig. 3C), the Chl/V_2_C NSs presented good transfection efficiency for cells (endocytosis), further confirmed by the ICP-MS analysis (Additional file 1: Fig. S7 A), which is helpful for high-effective therapeutics. Before investigating the anticancer effect of Chl/V_2_C NSs, the intracellular singlet O_2_ production ability was studied with a green hypoxia probe. The strong green fluorescence was observed in Chl/V_2_C NSs-treated cells under NIR irradiation (Fig. 3D), which suggested its good singlet oxygen generation ability, vital for hypoxia (cell death due to oxygen deficiency) in cancerous cells PDT.

**Fig. 3:** **A** Cytotoxicity of MCF-7 cells treated with PBS (pH 7.4,10 Mm), V_2_C, Chl and Chl/V_2_C (80 µg/mL), **B** CLSM of live/dead Calcein AM/PI staining of MCF-7 cells with different treatments, **C** CLSM images of Chl/V_2_C-treated MCF-7 cells for different time (scale bar = 10 μm), **D** Hypoxic level of PBS (pH 7.4,10 Mm) and Chl/V_2_C NSs (80 µg/mL) treated MCF-7 cells with N_2_ treatment irradiated with (+) /without (−) laser (scale bar = 100 nm). **E** MTT and **F** Calcein AM/PI staining anlysis of MCF-7 cells with different treatments

To comprehensively study the tumor cell killing ability of Chl/V_2_C NSs, the experiments were divided into eight groups as follows: (1) control PBS (pH 7.4,10 Mm) (2) laser 670 & 808 nm, (3) Chl/V_2_C NSs (4) Chl + 670 nm laser, (5) V_2_C NSs + 808 nm laser, (6) Chl/V_2_C NSs + 670 nm laser, (7) Chl/V_2_C NSs + 808 nm laser and (8) Chl/V_2_C NSs + 670 & 808 nm, respectively. Group 1, 2 and 3 showed negligible antitumor ability, and the increase in antitumor ability was observed for group 4–8 (group 4 < 5 < 6 < 7 < 8). The cell viabilities from group 1 to 8 was 99.2, 97, 92, 65, 50, 36, 20 and 1%, respectively (Fig. 3E). It indicated that the Chl and V2C could mediate PDT (group 4) and PTT (group 5). At the same time, the Chl/V_2_C NSs displayed enhanced therapeutic effects even under single laser irradiation (group 6 and group 7) due to the interaction between Chl and V_2_C. Under 670 and 808 nm laser irradiation, the Chl/V_2_C NSs prevented almost all tumors due to the synergistic effect. The results of Calcein-AM/PI dual-stained analysis were consistent with the cell viabilities analysis. (Fig. 3F). The intracellular quantification analysis of Chl/V_2_C at different intervals of time (1, 2, 3, 4 & 5 h), the quantification analysis of hypoxia with PBS and Chl/V_2_C, biodistribution and blood circulation of Mg concentrations measured with ICP-MS after injection of Chl/V_2_C to MCF-7 tumor-bearing mice (Mg being devoted by Chlorophyll) were investigated (Additional file 1: Figs. S7 and S8). The hypoxia condition in the tumor before and after treatment has been analyzed and shown in (Additional file 1: Fig. S9). These outcomes established the advanced in vitro antitumor capability of Chl/V_2_C NSs.

The article "Artificial photoactive chlorophyll conjugated vanadium carbide nanostructure for synergistic photothermal/photodynamic therapy of cancer" was retracted in 2023. Reasons: duplicated images; overlap with earlier publications; original data or images not available; unreliable data.

### In vivo anticancer performance of Chl/V_2_C NSs

The in vivo cancer therapeutic effect of Chl/V_2_C NSs was studied using mice exgrafed MCF-7 tumors. After intravenous inoculation of Chl/V_2_C NSs for 24 h, mice's main organs and tumors were collected to examine under ICP-MS (Fig. 4A). High accumulation of Chl/V_2_C NSs (∼30% ID/g) were detected due to the enhanced permeation retention effect and maintenance effect. High-level Chl/V_2_C NSs in the lungs and liver suggested that it could be fast cleared from the other main organs. The blood circulation in Chl/V_2_C NSs-treated samples were regulated in a two-compartment model. The half time was calculated to be 1.49 h, which highly stimulated and increased accumulation efficacy at the tumor site for therapy (Fig. 4B). The in vivo treatments were divided into 8 groups (n = 5): group (1) Control group PBS (pH 7.4, 10 mM), (20 mg/kg) (2) Laser 670 & 808 nm (3) Chl/V_2_C NSs (4) Chl + 670 nm, (5) V_2_C NSs + 808 nm, (6) Chl/V_2_C NSs + 670 nm, (7) Chl/V_2_C NSs + 808 nm and (8) Chl/V_2_C NSs, + 670 & 808 nm for 5 min laser (0.48 W cm^−2^). The weight of all the groups showed little difference, indicating the good biocompatibility of the Chl/V_2_C (Fig. 4C). The tumor volume (Fig. 4D and E) and tumor weight (Fig. 4F) of mice were monitored after treatment to estimate the therapeutic effect of each group. Group 1, 2, and 3 showed few therapeutic effects. Group 4 and group 5 displayed anticancer effects resulting from Chl-related PDT and V_2_C NSs-mediated PTT. The Chl/V_2_C NSs presented enhanced PDT (group 6) and PDT (group 7) compared to the Chl and V_2_C alone due to the interaction between Chl and V_2_C, which improved the high light absorption and energy conversion efficiency. Group 8 showed complete resistance to tumor growth, and the tumor almost disappeared after 12 days due to combined PTT & PDT. These results demonstrated the good in vivo anticancer ability of Chl/V_2_C NSs [30].

The article "Artificial photoactive chlorophyll conjugated vanadium carbide nanostructure for synergistic photothermal/photodynamic therapy of cancer" was retracted in 2023. Reasons: duplicated images; overlap with earlier publications; original data or images not available; unreliable data.

**Fig. 4:** **A** Biodistribution and **B** Blood circulation of V concentrations measured with ICP-MS after injection of Chl/V_2_C to MCF-7 tumor-bearing mice, **C** Body weight, **D** relative tumor volume curves, **E** digital images, **F** tumor weight analysis of MCF-7 tumor-bearing mice with different treatment (*n* = 5 mice per group)

### Biological biosafety analysis of Chl/V_2_C NSs

The hematoxylin–eosin (H&E) staining analysis of the key organs containing (spleen, kidney, lungs, liver, & heart) were conducted after the mice received treatment for two weeks. As shown in (Fig. 5A), no significant damage was detected in all main organs after comparing all groups, which illustrates the good in vivo biocompatibility of Chl/V_2_C NSs. (Fig. 5B) showed the H&E, TUNEL, and Ki—67 staining analysis, which indicated the tumor cells were not damaged in (1, 2 & 3) control groups. Groups 4 and 5 depicted fragmentary or little necrosis, while groups 6 and 7 demonstrated significant necrosis (Additional file 1: Fig. S10). The highest percentage of necrosis occurred in cancer cells of group 8, illustrating the excellent antitumor efficiency of Chl/V_2_C NSs. The in vivo toxicity was further studied after systemic administration of Chl/V_2_C NSs via intravenous injection. The normal blood biochemical profiling was done and multipurpose markers such as total bilirubin **(**TBL**),** aspartate aminotransferase (AST), alanine aminotransferase (ALT), blood urea nitrogen (BUN), globulin (GLOB), total protein (TP), creatinine (CREA), and albumin (ALB) were measured. (Fig. 5C-J) demonstrated that mice treated with Chl/V_2_C NSs exhibited abnormality compared to all groups, suggesting good compatibility of Chl/V_2_C NSs. [31]

**Fig. 5:** **A** The H&E staining analysis of the key organs, including lung, liver, kidney, spleen, and heart, obtained after treatments (scale bar = 100 nm). **B** Pathological changes in tumor tissues were demonstrated with H&E, TUNEL, and Ki67 staining (scale bar = 50 μm). **C**–**J** Biochemistry results of serum obtained from mice after injecting with PBS (pH 7.4,10 mM) and Chl/V_2_C (20 mg/kg) at 24 h. The blood intensities include TP, AST, ALT, BUN, TBL, ALB, and CREA

The article "Artificial photoactive chlorophyll conjugated vanadium carbide nanostructure for synergistic photothermal/photodynamic therapy of cancer" was retracted in 2023. Reasons: duplicated images; overlap with earlier publications; original data or images not available; unreliable data.

## Conclusion

In summary, we developed an optically active nanostructure of Chl/V_2_C NSs by modifying natural Chl derived from *Leptolyngbya JSC-1* extracts onto the surface of the V_2_C NSs for combined PTT and PDT. The interaction between organic Chl and metallic V_2_C sharply enhanced the light absorption and energy conversion efficiency. In this system, the Chl was used as a light-harvest antenna and PSs, while the V_2_C provided a large surface for Chl loading and acted as PTCAs. The Chl/V_2_C enabled O_2_ generation to relieve hypoxic TME and displayed improved ROS species generation ability, including ^1^O_2_, ·OH and·O_2_^−^ for PDT. It also showed a PTCE high of 78%, superior to most of the previous 2D PTCAs. We demonstrated the advanced anticancer effect of the Chl/V_2_C both in vitro and in vivo, and the tumor growth was inhibited entirely after Chl/V_2_C-mediated combined PTT/PDT. Our results suggest that the Chl/V_2_C holds excellent promise for phototherapy and paves a new way to design artificial optical nanostructure for phototherapy rationally.

## Supplementary Information

**Additional file 1: Scheme S1**. Schematic elastration of ROS production mechanism. **Figure S1**. A, B and C The comparison of standard and extracted Chlorophyll (Chl) and confirm the loading Chl on V2C. Scheme S1: The ROS production mechanism scheme. **Figure S2**. Zeta potential analysis. **Figure S3**. A, B and C: The EDX analysis. **Figure S4**. A, B and C: Loading efficiency of of chlorophyll (Chl) on V2C SNs. (B) temperature increasing (Chl) and (C) oxygen generation measurement with various loading concentration of Chl. **Figure S5**. A, B: To measure the photothermal conversion efficiency of Chl/V2C NSs. **Figure S6**. Cell viabilities performance of Chl/V2C for different cell lines. **Figure S7**. A, B: The intracellular and hypoxia quantification analysis of Chl/V2C. **Figure S8**. A, B: Biodistribution and) Blood circulation of Mg concentrations measured. **Figure S9**. Hypoxia analysis of tumours untreated and treated with Chl/V2C SNs. **Figure S10**. Statistical analysis Ki-67 A and B TUNEL assessment of all the tumors.

## Data Availability

The current study data are available from the corresponding author on reasonable request.

## Abbreviations

PTT: Photothermal therapy
PTT: Photodynamic therapy
Chl: Chlorophyll
V_2_C: Vanadium carbide
PSs: Photosensitizers
2D: Two-dimensional
TBL: Total bilirubin
AST: Aspartate aminotransferase
ALT: Alanine aminotransferase
BUN: Blood urea nitrogen
GLOB: Globulin
TP: Total protein
CREA: Creatinine
ALB: Albumin
TME: Tumor microenvironment
nm: Nano meter
μm: Micro meter
TEM: Transmission electron microscopy
EDX: Energy dispersive X-ray spectroscopy spectra
FTIR: Fourier transform infrared spectroscopy
DLS: Dynamic light scattering
CLSM: Confocal laser scanning microscopy
